The article "Analysis of Clinical Manifestations and Imaging of COVID-19 Patients in Intensive Care" was published in 2022. Journal: Contrast Media Mol Imaging.

# Analysis of Clinical Manifestations and Imaging of COVID-19 Patients in Intensive Care

**DOI:** 10.1155/2022/9697285

**Published:** 2022-06-23

**Authors:** Lihong Li, Yongwei Yao, Xiaofei Feng, Lingling Chen, Rui Wu, Yuejin Chang, Qiaoqin Lou, Jinbo Pan, Zhangli Wang

**Affiliations:** ^1^The Second Affiliated Hospital of Zhejiang Chinese Medical University, Xinhua Hospital of Zhejiang Province, Hangzhou 310005, China; ^2^Oncology Department, Hangzhou Third Hospital, Hangzhou 310009, China; ^3^Emergency Department, Hangzhou Third Hospital, Hangzhou 310009, China; ^4^Nephropathy Department, Hangzhou Third Hospital, Hangzhou 310009, China; ^5^ICU, Hangzhou Third Hospital, Hangzhou 310009, China; ^6^Hebei Yanda Hospital, Langfang 065200, China

## Abstract

**Objective:**

The study aims to summarize and analyze the clinical and CT findings of severe COVID-19 patients.

**Methods:**

From February 11 to March 31, 2020, 61 COVID-19 patients in intensive care in the E1-3 ward of Tongji Hospital were analyzed retrospectively.

**Results:**

The main clinical manifestations were cough, expectoration in 56 cases (91.8%), shortness of breath, chest tightness in 48 cases (78.7%), fever in 61 cases (100%), muscle ache and weakness in 40 cases (65.6%), diarrhea or vomiting in 8 cases (13.1%), and headache in 4 cases (6.6%). After admission, the leukocyte count was normal in 40 cases (57.7%), higher in 9 cases (15.4%), and lower in 12 cases (26.9%). The lymphocyte count decreased in 53 cases (86.9%). CRP was increased in 29 cases (47.5%); PCT was increased in 15 cases (24.6%); ESR was increased in 38 cases (62.3%); D-dimer increased in 39 cases (63.9%); ALT/AST increased in 40 cases (65.6%); CK/CK-MB increased in 8 cases (13.1%); troponin I increased in 6 cases (9.8%); NT-proBNP increased in 35 cases (57.4%); IL-1 increased in 5 cases (8.2%); IL-2 receptor increased in 28 cases (45.9%); IL-6 increased in 23 cases (37.7%); IL-8 increased in 15 cases (24.6%); IL-10 increased in 12 cases (19.7%); and NTF increased in 22 cases (36.1%). The chest CT images showed that 38 cases (65.5%) of right lung lesions were more extensive than those of left lung lesions, 20 cases (34.5%) of left lung lesions were more extensive than those of right lung lesions, 42 cases (72.5%) of lower lobe lesions were more extensive than those of upper lobe lesions, 6 cases (10.3%) of upper lobe lesions were more extensive than those of lower lobe lesions, and 10 cases (17.2%) of upper and lower part lesions were roughly the same. Ground-glass opacity (GGO) was found in 12 cases (20.7%); GGO with focal consolidation in 38 cases (65.5%); small patchy edge fuzzy density increased in 24 cases (41.4%); large consolidation in 20 cases (34.5%); reticular or fibrous cord in 54 cases (93.1%); and air bronchogram in 8 cases (13.8%).

The article "Analysis of Clinical Manifestations and Imaging of COVID-19 Patients in Intensive Care" was published in 2022. Journal: Contrast Media Mol Imaging.

**Conclusions:**

COVID-19 patients in intensive care have no specific clinical manifestation and CT findings. However, analysis and summary of relevant data can help us assess the severity of the disease, decide the timing of treatment, and predict prognosis.

## 1. Introduction

As of April 14, 2020, coronavirus disease 2019 (COVID-19) has spread across 185 countries/regions, infected more than 1.9 million people, and killed 120 thousands of people. To this day, COVID-19, which is “not very impressive,” can cause such a great “lethality” in the progress of science and technology and the highly developed medical science. The reason is that we do not know enough about the “little virus” or have enough imagination about its impact. All we can do now is to know as much as we can about it. COVID-19 is a new type of severe pneumonia. We have collected clinical manifestations and CT imaging findings of 61 COVID-19 cases in intensive care.

## 2. Materials and Methods

### 2.1. Objects

From February 11, 2020 to March 31, 2020, 61 adult patients in intensive care were admitted to the ward E1-3 of Tongji Hospital. Forty-five patients were selected from community isolation clinic and hospital fever clinic on February 11, 2020, and the rest 16 cases were transferred from the designated hospital. Sixty-one patients were confirmed by diagnostic criteria of China COVID-19 treatment (fifth, sixth, and seventh Edition). Detection novel coronavirus nucleic acid positive by RT-PCR in specimens (mouth/nasopharyngeal swabs), and/or COVID-19 specific anti-IgM and anti-IgG were positive in serum samples. At the same time, all patients at the time of admission have any of the following conditions: (1) shortness of breath and respiratory rate (RR) ≥ 30 times/min; (2) at rest, refers to oxygen saturation ≤93%; and (3) arterial blood oxygen partial pressure (PaO2)/oxygen concentration (FiO2) ≤ 300 mmHg, which are the COVID-19 cases in intensive care unit. Among them, 6 patients had one of the following conditions during hospitalization: (1) respiratory failure, and mechanical ventilation was required; (2) shock occurred; and (3) combining other organ failures required ICU monitoring treatment, and the diagnosis was severe COVID-19. Of the 61 patients included in the study, male 32 and female 29, aged 24–83, mean age (58.52 ± 1.67), 18 patients with hypertension, 11 patients with diabetes or stress hyperglycemia, and chronic heart disease 9 cases, COPD 3 cases, gout 3 cases, chronic kidney disease 2 cases, and hematological malignancy 1 case.

The article "Analysis of Clinical Manifestations and Imaging of COVID-19 Patients in Intensive Care" was published in 2022. Journal: Contrast Media Mol Imaging.

### 2.2. Treatment Plan

Treatment mainly covers six aspects: First, choose the appropriate oxygen therapy according to the degree of dyspnea of the patient. Most patients use a dual-cavity nasal catheter to inhale oxygen. The oxygen flow is 3–5 L/min. The target refers to oxygen saturation ≥93%, and a noninvasive ventilator is immediately used when unable to meet the needs. Second, the antiviral treatment plan is determined and Abidor 200 mg, 3 times a day or lopinavir/ritonavir 200 mg/50 mg/capsule, 2 capsules each time, 2 times a day. Two critically ill patients used 5 million units of *α*-interferon in combination with daily nebulized inhalation, ribavirin 500 mg, and intravenous infusion twice daily. The duration of antiviral treatment is 10 days. Third, based on the patient's respiratory symptoms and changes in CT imaging, we decide whether to use glucocorticoids. If the patient has shortness of breath and the respiratory rate is greater than 30 breaths per minute, when the CT imaging shows that the exudation is the main change, you can optionally use methylprednisolone 40–80 mg intravenous drip and evaluate it again after 5 days. It should either be used or stopped directly. Fourth, based on the treatment of the patient's symptoms, acetaminophen is administered when the body temperature (frontal temperature) is ≥102.2°C, bronchial spasm relief drugs and acetylcysteine tablets 0.6 g orally, 2 times a day, and when the cough and sputum are obvious 0.3 g of acetylcysteine solution is used for inhalation or 3 times a day. Fifth, nutrition support is strengthened to ensure that the daily calorie intake of the patient is greater than 35 Kcal/kg and infusion of 20% human serum albumin solution makes the patient's serum albumin level greater than 30 g/L. Sixth, the possibility of secondary bacterial or fungal infections is assessed.

### 2.3. Observation Indicators

Onset time, primary symptoms, epidemic history, nucleic acid testing (NAT) results, CT imaging results, and medicine treatment were taken into account before admission. Blood routine, CRP, PCT, ESR, liver enzyme, myocardial enzyme spectrum and troponin I, NT-proBNP, D-dimer, inflammatory factors, and chest CT imaging were detected irregularly.

## 3. Results

### 3.1. Prognosis

Of the 61 patients, 3 died after tracheal intubation and treated with a ventilator and 1 patient with acute hematological malignancies died of secondary multidrug resistant bacteria (CRE) bloodstream infection The symptoms of the remaining patients disappeared or were significantly alleviated. The chest CT scan showed obvious absorption of the lesion, and the patient was discharged after retesting negative NAT.

### 3.2. Clinical Features

Sixty-one patients were local Wuhan personnel, and most of them had a clear history of epidemiological contact (77%), with 61 cases of fever (100%) as the first symptom, 56 cases of cough and expectoration (91.8%), 48 cases of shortness of breath and chest tightness (78.7%), muscle soreness and fatigue in 40 cases (65.6%), diarrhea or vomiting in 8 cases (13.1%), and headache in 4 cases (6.6%). At admission, 15 patients had a course of ≤7 d, 23 patients from 8–14 d, and 23 patients >14 d. Before admission, all patients underwent different degrees of medicine treatment, including 3 cases of Abidor, 8 cases of ribavirin, 15 cases of oseltamivir, 10 cases of glucocorticoids, 28 cases of antibiotics, 57 cases of antipyretics and, 61 cases of Chinese herbal medicine preparation.

The article "Analysis of Clinical Manifestations and Imaging of COVID-19 Patients in Intensive Care" was published in 2022. Journal: Contrast Media Mol Imaging.

After admission, 40 cases of normal white blood cell count (57.7%) were checked, 9 cases (15.4%) were higher than normal, and 12 cases (26.9%) were lower than normal. The lymphocyte count decreased in 53 cases (38.5%). CRP increased in 29 cases (57.7%); PCT increased in 15 cases (24.6%); the erythrocyte sedimentation rate increased in 38 cases (62.3%); the D-dimer test increased in 39 cases (63.9%); ALT/AST increased in 40 cases (65.6%); CK/CK-MB increased in 8 cases (13.1%); troponin I increased in 6 cases (9.8%); NT-proBNP increased in 35 cases (57.4%); IL-1 increased in 5 cases (8.2%); IL-2 increased in 28 cases (45.9%); IL-6 increased in 23 cases (37.7%); IL-8 increased in 15 cases (24.6%); IL-10 increased in 12 cases (19.7%); and NTF increased in 22 cases (36.1%), which are shown in Table 1.

### 3.3. Imaging Features

Of 61 COVID-19 patients, 3 patients were in critical condition after admission, unable to complete chest CT examination, and died after being transferred to ICU. The remaining 58 patients completed chest CT examination. There were 38 cases (65.5%) with a wider range of right lung lesions than left lung lesions and 20 cases (34.5%) with a wider range of left lung lesions than right lung lesions. There were 42 cases (72.5%) with lower lobe lesions than upper lobe lesions, and 6 cases (10.3%) with upper lobe lesions than lower lobe lesions are shown in Table 2.

From the picture, 58 COVID-19 patients showed one or more of the following signs: ground-glass opacity (GGO) was found in 12 cases, with subpleural distribution (Figures 1(a) and 1(b)); GGO merger in 38 cases of focal consolidation (Figures 1(c) and 1(d)); 24 cases with increased patch density of small patchy edges (Figures 1(c) and 1(f)); large consolidation of sheets in 20 cases(Figures 1(e) and 1(g)); 54 cases with grid-like or fibrous strips (Figures 1(c)–1(e)); and 8 cases with air bronchial signs (Figure 1(c)).

The article "Analysis of Clinical Manifestations and Imaging of COVID-19 Patients in Intensive Care" was published in 2022. Journal: Contrast Media Mol Imaging.

## 4. Discussion

COVID-19 is caused by the severe acute respiratory syndrome coronavirus-2 (SARS-CoV-2) [1], and it is obviously different from severe acute respiratory syndrome (SARS) and the Middle East respiratory syndrome (MERS) that were popular several years ago [2]. Similarly, it is different from viral pneumonia such as influenza virus pneumonia, parainfluenza virus pneumonia, influenza A virus pneumonia, avian influenza virus pneumonia, adenovirus pneumonia, respiratory syncytial virus pneumonia, and cytomegalovirus pneumonia [3–6]. At the beginning of the epidemic in Wuhan, everyone could only think of it as an unexplained pneumonia. At present, it is known that COVID-19 is mainly spread through respiratory droplets and close contact and there is a possibility of aerosol transmission when exposed to a high concentration of aerosol for a long time in a relatively closed environment. Most CoVs share a similar viral structure and infection pathway [7–10]. COVID-19 is highly contagious and long-term latent, and the population is generally susceptible, which makes it difficult to control once it breaks out. Moreover, in the early stage of the disease, there is no effective treatment, and there is a considerable possibility that it will progress to severe disease, affecting whether it is elderly or young [11, 12]. Of the 61 cases of severe new coronary pneumonia we treated, only 27 were older than 60 years, but 46 patients had a disease course of more than 7 days. Although they all received medical treatment, they were treated based on their lack of understanding of the disease at that time. Owing to limited medical resources, the effect of treatment is not ideal. This situation was very common in the early days of the outbreak in each country, and a large number of serious patients requiring hospitalization appeared, including many young people. The clinical manifestations of these people with severe new coronary pneumonia are actually not specific. We cannot identify COVID-19 by symptoms such as fever, cough, shortness of breath, chest tightness, muscle aches, fatigue, and diarrhea. We also did not observe symptoms of loss of smell or taste. However, some of these symptoms are important in determining the severity and prognosis of the disease. The 61 patients included in the study had symptoms of fever at the beginning of the disease, but after a long period of time, 11 patients still had symptoms of fever at admission. These people included all 6 patients who required noninvasive ventilator treatment, including 3 of them who died after being transferred to ICU. Similarly, shortness of breath or the increased breathing rate and feeling chest tightness are also an important red flag. Therefore, 38 of the 61 patients we admitted had shortness of breath and chest tightness. When the symptoms of shortness of breath cannot be alleviated by oxygen therapy or symptomatic treatment, special vigilance is required. Our experience is to intervene early and actively intervene. There are 2 critically ill patients who passed the most difficult stage through our early-rising noninvasive ventilator treatment and avoided being transferred to ICU. Some of these patients did take Chinese herbal medicine. However, because the patients were in the early stage of emergency treatment, we were unable to take it regularly, nor did we carry out the role of Chinese herbal medicine in the treatment of critically ill patients. Temperature and respiratory rate, or fever, and shortness of breath are very easy to get, and they are very useful clinical manifestations. The rest of the symptoms are of limited significance.

The article "Analysis of Clinical Manifestations and Imaging of COVID-19 Patients in Intensive Care" was published in 2022. Journal: Contrast Media Mol Imaging.

The total number of peripheral blood leukocytes in patients with COVID-19 is normal or reduced, and the lymphocyte count is reduced. In some patients, ALT/AST, CRP, ESR, D-dimer, NT-proBNP, IL-1, IL-2 receptor, IL- 6. IL-8, IL-10, and NTF increased. In critically ill patients, troponin, IL-2 receptors, IL-6, and NTF will increase significantly, which means the advent of inflammatory storm. This is an important time point for us to start some special treatments, including the use of glucocorticoids, infusion recovery period plasma, and CRRT. White blood cell count, CRP, and PCT of patients with severe new coronary pneumonia can increase simultaneously as one of the basis for judging secondary bacterial infection.

We must recognize that chest CT imaging plays an important role in the diagnosis, treatment, and follow-up of COVID-19. Imaging examination revealed that most patients showed bilateral GGO on CT scans [13, 14]. CT is a sensitive examination method, which can be applied to make an early diagnosis and for evaluation of progression, with a diagnostic sensitivity and accuracy better than that of nucleic acid detection [15]. Therefore, we try to complete the patient's CT scan as much as possible. Sixty-one cases of COVID-19 were admitted to the intensive care, and we can only get the results of the CT image before the admission and lack of its imaging data. After admission, we improved the chest CT examination of 58 patients. Based on the results of chest CT scans of 58 patients with severe COVID-19 included in the study, the CT imaging findings were summarized as follows: the lesions have multiple lung segments and lobes, involving both sides, with a wider range. It is more common under the pleura; most of the lesions are grid or fibrous cord shadow, patchy density increase shadow, GGO with consolidation shadow, and segmental or subsegmental GGO lesions can also be seen, and air bronchial signs can be seen in the lesion or thickened blood vessels. These imaging findings are basically consistent with the pathological anatomical results of COVID-19. The bronchi are covered with mucus and bleeding exudates. Histological examination revealed bilateral diffuse alveolar injury with mucous exudation of cell fibers and a large amount of pulmonary interstitial fibrosis with part transparent degeneration, and pulmonary hemorrhagic infarction. But we found two interesting phenomena. The severity of the disease in the right lung and lower lobe of patients with severe COVID-19 is more serious, which may be related to the different proportions of ventilated blood flow in different parts.

The article "Analysis of Clinical Manifestations and Imaging of COVID-19 Patients in Intensive Care" was published in 2022. Journal: Contrast Media Mol Imaging.

## 5. Conclusion

In summary, the clinical manifestations of patients with severe COVID-19 are not specific to the chest CT manifestations. The assessment of the disease requires a comprehensive analysis of relevant symptoms, signs, and laboratory data so as to help us judge the severity of the disease and decide timing of treatment and assess the prognosis.

## Figures and Tables

**Figure 1:** Characteristics of lung CT manifestations in patients with COVID-19.

**Table 1:** Clinical feature analysis results of 61 COVID-19 patients.

Characteristics		*n*	Ratio (%)
Symptoms	Epidemiological exposure	47	77.0
	Fever	61	100.0
	Cough	56	91.8
	Shortness of breath	48	78.7
	Muscle soreness	40	65.6
	Diarrhea/vomiting	8	13.1
	Headache	4	6.6

Course of disease	≤7 d	15	24.6
	8–14 d	23	37.7
	>14 d	23	37.7

Medicine treatment	Chinese herb	61	100.0
	Abidor	3	4.9
	Ribavirin	8	13.0
	Glucocorticoids	10	16.0
	Antipyretics	57	93.0
	Antibiotics	28	45.9
	Oseltamivir	15	115.8

Laboratory examination	WBC count		
	Normal	40	57.7
	Higher	9	15.4
	Lower	12	26.9
	Lymphocyte count		
	Decreased	53	86.9
	CRP		
	Increased	29	47.5
	PCT		
	Increased	15	24.6
	ESR		
	Increased	38	62.3
	D-dimer	39	63.9
	ALT/AST	40	65.6
	CK/CK-MB		
	Increased	8	13.1
	Troponin I		
	Increased	6	9.8
	NT-proBNP	35	57.4
	IL-1		
	Increased	5	8.2
	IL-2		
	Increased	28	45.9
	IL-6		
	Increased	23	37.7
	IL-8		
	Increased	15	24.6
	IL-10		
	Increased	12	19.7
	NTF		
	Increased	22	36.1

**Table 2:** Chest CT examination analysis results of 61 COVID-19 patients.

Characteristics		*n*	Ratio (%)
CT scan	Performed	58	95.1
	Not performed	3	4.9

Affected lobe	Right	38	65.5
	Left	20	34.5
	Lower	42	72.5
	Upper	6	10.3

Signs	GGO	12	20.7
	Focal consolidation	38	65.5
	Lung consolidation	20	34.5
	Grid-like or fibrous strips	54%	93.1
	Air bronchial signs	8	13.8

The article "Analysis of Clinical Manifestations and Imaging of COVID-19 Patients in Intensive Care" was published in 2022. Journal: Contrast Media Mol Imaging.

## Data Availability

The datasets used and/or analyzed during the current study are available from the corresponding author on reasonable request.

## Abbreviations

COVID-19: Coronavirus disease 2019
CT: Computed tomography
GGO: Ground-glass opacity
ICU: Intensive care unit
NAT: Nucleic acid testing.
